This article has been retracted.

# Preparation of Bismuth Tungstate Nanomaterials with Different Morphologies and Their Effect on Exercise Rehabilitation of Patients with Lumbar Disc Herniation

**DOI:** 10.1155/2022/1397896

**Published:** 2022-01-07

**Authors:** Xiao Ma, Dezhi Kong, Zihui Chang

**Affiliations:** ^1^School of Physical Education, Liaocheng University, Liaocheng, Shandong 252000, China; ^2^Department of Physical Education, Hainan Medical College, Haikou, Hainan 571199, China; ^3^Liaocheng People's Hospital, Liaocheng, Shandong 252000, China

## Abstract

It is understood that the effect of exercise rehabilitation drugs in patients with lumbar disc herniation is poor. Some studies have shown that bismuth tungstate nanomaterials with certain morphology can treat the exercise rehabilitation of patients with lumbar disc herniation. In order to help patients with lumbar disc herniation to a certain extent, in this paper, bismuth tungstate nanomaterials with different structures and morphologies were prepared by hydrothermal method, and viscous tungsten nanomaterials with different structures and morphologies were prepared by adjusting the pH value of the solution and the concentration of CTAB. In this paper, the structure and morphology of tungsten samples with different structure and morphology were characterized by CTAB X-ray (XRD) deflection and FESEM. It was found that the morphology of the samples changed after adding 0.02 mol/L surfactant CTAB in the reaction system, and when the concentration of CTAB was 0.04 mol/L, the nanotubes were stacked together under the action of surfactant. When the concentration of CTAB increased to 0.06 mol/L, the self-assembled nanocomposites tended to be petal like.

## 1. Introduction

Lumbar disc herniation (LDH) refers to the rupture of part or all of the lumbar disc due to various reasons (degeneration, disorder, injury, etc.). The spinal nerve root and cauda equina are ruptured, irritated or compressed, and protrude back, causing backache and leg pain or bladder and rectal dysfunction, that is, low back pain with sciatica or secondary spinal dysfunction. Among them, lactic acid is one of the common reasons for aggravating low back pain.

Tungstate nanomaterials have good application prospects in the fields of foaming materials, optical fibers, light sources, microwave applications, water sensors, photocells, semiconductor materials, magnetic devices, and the treatment of disc herniation. In the past few years, tungstate nanomaterials have become a hot research topic. Bismuth tungstate (Bi_2_WO_6_) has photocatalytic activity under visible light with wavelength over 420 nm. Bismuth tungstate (Bi_2_WO_6_) is a photocatalyst with visible light, which can decompose organic pollutants in water under the excitation of visible light. Its modification can not only make the catalyst have some special properties, but also improve its photocatalytic degradation performance. It is also used for the treatment of lumbar disc herniation. Bi_2_WO_6_ has a narrow restricted area width (about 2.7 eV). It can be excited by visible light and has high catalytic activity under visible light. As a new photocatalytic material, it has attracted more and more attention. The study of Bi_2_WO_6_ in the treatment of lumbar disc herniation is the study of its catalytic effect under different morphology on the treatment of lumbar disc herniation, which has very important medical value in the treatment of lumbar disc herniation and drug research and development.

The overuse and persistence of antibiotics will lead to various environmental hazards and health risks. Therefore, accurate sensors are needed to determine their presence. In this work, Munawar et al. proposed a quality sensitive sensor for detecting rifampicin. They chose this molecule because it is an important antibiotic for tuberculosis, and tuberculosis is one of the main causes of death worldwide. Here, a simple in situ synthesis mechanism can be used to prepare bismuth tungstate nanocomposite reinforced carbon nanotubes in a clear nanosheet shape. The synergy of the complex thus formed shows a high affinity for rifampicin compared with the single component of the complex, but the experimental operation is a little complex [1]. Bismuth tungstate (Bi_2_WO_6_) has many interesting properties and has been the focus of research in many fields, especially photocatalysis. Yuan et al. successfully synthesized ultrathin nanosheets with crystalline amorphous composite phase and assembled ordered Bi_2_WO_6_ by one-step hydrothermal method. The composition, morphology, and microstructure were characterized by X-ray diffraction (XRD), X-ray photoelectron spectroscopy (XPS), field emission scanning electron microscopy (FESEM), and high-resolution transmission electron microscopy (HRTEM). It has good reproducibility and long-term stability (more than 50 days). The performance of Bi_2_WO_6_ is better than the existing sensing platform based on Bi_2_WO_6_ and most other advanced sensing platforms, but it has not been applied in large-scale enclosure [2].

In this experiment, bismuth tungstate nanomaterials were prepared by hydrothermal method, and the preparation process is simple. By changing the hydrothermal conditions, the particle size and morphology of the product can be controlled so as to change the properties of the product. In this paper, hydrochloric acid is used instead of lactic acid, which makes people ache. The catalytic effect of bismuth sodium tungstate with different morphology on hydrochloric acid is analyzed and discussed. The relevant research and discussion are carried out for different pH values and CTAB concentrations. Among them, when the pH value is 9 or the CTAB concentration is 0.08 mol/L, bismuth tungstate sodium formed has the best catalytic effect on hydrochloric acid at most. A new field of research has been made on the treatment of lumbar disc herniation and rehabilitation effect with bismuth tungstate nanomaterials.

## 2. Proposed Method

### 2.1. Etiology of Lumbar Disc Herniation

#### 2.1.1. Retrogressive Change

Usually, after the age of 20, the median disc begins to degenerate, and obvious degeneration occurs after the age of 30, leading to disc degeneration. By compressing and stimulating the nerve root and salivary sac, inflammatory transmitters are produced, and the pain is caused by the role of sinus nerve injury sensor. Compressing the nerve root can lead to numbness of lower limbs on the corresponding side, radioactive pain, and numbness of lower legs and dorsum of feet, which is the most common cause of low back pain in the elderly.

#### 2.1.2. Injury and Strain

It mainly includes acute lumbar sprain, chronic lumbar muscle injury, spine and distal joint injury, and the third lumbar transverse process syndrome. According to foreign reports, the causes of low back pain caused by trauma are 30% to 70%; low back pain is related to the circulatory load caused by persistent spinal cord spasm and delay of overstimulation, repeated high-frequency and high-speed spinal movement [3]. When the strength of the lower back muscle is weakened, the spine is overloaded, which is easy to cause acute dislocation of the spine, and the poor posture of the waist can cause chronic muscle injury. As a result, the stability of the media decreased, leading to lumbar disc herniation.

### 2.2. Biomechanics and Lumbar Disc Herniation

The excessive displacement of some parts of the spine under the action of external forces will cause back pain. Long sitting and long staying time will increase the load of the media disk and cause the disk to protrude. The patients with lumbar degenerative change, spondylolisthesis, or instability are mostly seen in the middle-aged and old people, which leads to recurrent lower back attack and leg pain. The main factors causing back pain are the decrease of spinal cord stability and muscle strength.  Figure 1 shows the effect of excessive displacement of some parts of the spine.

The stability of the spine of the three-subsystem model refers to the deformation of the spine under the ability load to maintain the normal spine. The central nervous system subsystem uses neural circuits to control muscle contraction time, sequence, and intensity. When disease occurs in any of the three subsystems, the other two subsystems will temporarily compensate for the loss of function so as to maintain lumbar balance [4, 5]. When the passive support system and central nervous system develop diseases, it is difficult to recover their functions through nonprofessional treatment. Only active support subsystem can recover its function through muscle training to maintain back balance.

Since 2000, sports medicine experts have paid more and more attention to the stability and stability of core muscles. Core stability is the ability of the complex system of the waist, pelvis, and thigh to control the curvature and recovery of the spine [6]. The core of the muscle consists of muscles around the spine and all the limbs of the body. It can stabilize the activities of the spine, pelvis, and joints and let people complete different actions. It can be divided into three types: global stable muscle, local stable muscle, and general exercise muscle. Completely stable muscle group: this muscle group belongs to the most superficial muscle group, which makes dynamic bending and expansion more intense. It includes good abdominal area, external dislocation, anterior abdominal dislocation, spiral erection, and thigh and hip. The local stable muscle group refers to the deeper muscle group, which can make it have greater static local stability and adjust the posture of spine. It includes multiskeletal muscle, transverse abdominal muscle, psoas major muscle, quadratus medius muscle, posterior internal flexor, and diaphragm and pelvis muscle. The main cause of spinal cord decline is local stable muscles, which are deep muscle groups and perfect spine posture. Among them, multiple muscle atrophy is the cause of lower back muscle weakness. Abdominal muscle is the competitive muscle of paracerebrum muscle. In patients with congenital abdominal muscle hypoplasia, scoliosis may be caused by imbalance.

### 2.3. Treatment of Lumbar Disc Herniation

The treatment of lumbar disc herniation mainly starts from surgical treatment and nonsurgical treatment. Nonoperative treatment methods mainly include basic treatment, self-function exercise, lumbar core stable muscle group training, attraction, physical therapy factors, medical treatment, psychological intervention, and traditional Chinese medicine [7]. The use of surgical treatment must follow the surgical indications. Doctors are required to choose different treatment methods for different patients and formulate formal treatment plans. The plan is well planned and reasonably arranged. Different measures are adopted in different stages from symptom relief, cure to recovery. The selected treatment method shall be adjusted in time according to the condition of the patient, and the psychological state of the patient shall be paid attention to at the same time. Nonoperative treatment is generally the first onset. In principle, nonsurgical treatment should be used first, unless the condition is more serious. The requirement is that if the symptoms are mild, the course of disease may last longer, but the nucleus pulposus is mostly prominent rather than prolapsed, which is easy to cure. Patients with unclear diagnosis are often confused by a variety of diseases, so it is difficult to make a clear diagnosis early. They need to take corresponding inspection measures during nonsurgical treatment, observation, and examination. Those whose general or local conditions are not suitable for operation mainly refer to elderly and frail patients, or those with other lesions in the operation area. Others include contraindications to surgery or anesthesia, or patients who refuse surgery.

#### 2.3.1. Basic Treatment

Basic treatment should be the first choice for the treatment of lumbar disc herniation. After regular basic treatment, most patients will get satisfactory results.

*(1) Bed Rest*. In the acute phase of pain, you need to rest in bed for a week. The pressure of the middle back disc should have the maximum displacement position in the sitting position, the maximum displacement position in the upright position, and the maximum displacement position in the immersion position. Braking may reduce the compression of the intermuscular disc and the tension of the intermediate link of the intermediate disc. The good muscle stability of the waist, ligament, and spine can also be maintained by eliminating edema, accelerating the reduction of inflammation caused by repeated movements of spinal nerve during the operation and avoiding walking or exercise for nerve root stimulation. We usually rest on mattresses of medium hardness.

*(2) Medication*. There are different reasons for choosing drugs. Commonly used drugs include nonsteroidal anti-inflammatory drugs, calcium or estrogen supplements, vitamin B, glucocorticoids, opioid analgesics, muscle relaxants, and antidepressants. Nonsteroidal anti-inflammatory drugs mainly have antipyretic, analgesic, and anti-inflammatory effects, but also inhibit platelet aggregation and tumor occurrence, development, and metastasis. Glucocorticoids are mainly involved in the metabolism of sugar, fat, and protein, as well as other pharmacological effects, such as anti-inflammatory, immunosuppressive, and antiallergic. In addition, the unique Chinese medicine preparation is oral, local fumigation, external application, iontophoresis, etc. It also has the effects of analgesia, promoting blood circulation and removing blood stasis. In a word, it should follow the principle of individualized medication.

#### 2.3.2. TCM Therapy

Observing the clinical effect of traction orthopedic treatment on lumbar disc herniation, Chinese herbal fumigation includes agrimony, 100 mu grass, xylene, Caifeng, ginseng, and Lutong [8].

#### 2.3.3. Rehabilitation Treatment

The purpose of rehabilitation treatment of lumbar disc herniation is to reduce or even eliminate clinical symptoms through comprehensive and coordinated application of various measures, to maintain the good ability of daily life activities, and finally to return to society and improve the quality of life [9, 10]. The main treatment measures are as follows:

*(1) Lumbar Traction.* Lumbar traction is the first choice for nonsurgical treatment of lumbar disc herniation. Its mechanism is that the separation of mechanical forces changes the relative position of the center of the middle disc and the back of the fiber and changes the interface between the middle disc and the nerve so as to reduce the nerve pressure [11]. In recent years, clinical three-dimensional mechanical attachment, such as spinal cord vibration sliding, utilizes body weight traction and works with transverse wavelengths to fully extend the spine. It has a good effect on lumbar disc herniation, lumbar lateral disorder, and lumbar motion, especially for the elderly. It is a safe, less painful, and simple treatment.

*(2) Physical Factor Therapy.* The application of physical factors in clinic has a long history, mainly including physical factors such as sound, light, electricity, and magnetism. The main curative effects are to promote blood circulation, improve the nutrition of local tissues, improve the vitality of cell tissues, accelerate the absorption or elimination of pathology and metabolites, promote wound healing, and eliminate inflammation. It can inhibit and excite the nervous system. The former can calm, relieve pain and relieve spasm, and inhibit the pathological excitation focus in the cerebral cortex; the latter helps to treat diseases such as nerve paralysis, perceptual disorder, muscle weakness, and muscle atrophy. It can also improve the regulation ability of body temperature and cardiovascular system and enhance the ability to resist diseases and adapt to environmental changes. It has certain curative effect on low back pain caused by various reasons [12]. At present, the commonly used conventional treatment methods are cold compress, which is suitable for the acute stage of various injuries; wax compress, which is suitable for the repair stage of various injuries; pulse electrotherapy, which was found in the clinical observation of patients with low back pain treated by computer intermediate frequency treatment instrument as early as the nineties, the computer intermediate frequency treatment group has significant curative effect, rapid effect, and good analgesic effect. Ultrashort wave therapy is used for the treatment of lumbar disc and foot. It has anti-inflammatory and analgesic effects, can effectively relieve pain, improve spinal cord dysfunction, and restore daily life activities. For the acute myogenic mass caused by irreversible syndrome, continuous low-level hyperthermia can significantly reduce the intensity of pain, reduce the pain, and improve the efficacy of the obstacles; the clinical trials of ultrasound treatment confirmed that the use of ultrasound penetration drugs to treat soft tissue injury. Exactly, there are microwave therapy, magnetic therapy, and so on. They have good results. Among them, intermittent electrotherapy and excessive infrared wave therapy are widely used in clinical work because of their simple operation, with definite curative effect, safety, simplicity, economy, and practicality.

*(3) Exercise Therapy.* Movement is the application of bio mechanical principle, using active or passive movement to improve patients' dysfunction. The purpose of the treatment of low back pain is to improve the range of motion of the spine, relieve the pain, and strengthen the strength of the back and abdominal muscles so as to maintain the stability of the spine and enhance the ability of daily life.

*(4) McKenzie's Treatment Technology.* The technology comes from the West and was founded by McKinsey, a New Zealand physiotherapist. It is mainly used for the treatment of cervical and lumbar diseases. Mackenzie's mechanical diagnosis and treatment methods have been used for many years in foreign countries. It is a commonly used method for physiotherapists to treat low back pain [13, 14]. The principle of treatment is to reduce the pressure of the central disc on the lumbar joint during the spinal stretch movement so that the protruding nucleus pulposus moves forward so as to reduce the pressure on the nucleus pulposus of the extension of the peripheral nerve root and to reduce symptoms and achieve the purpose of treatment. In McKenzie's processing technology, centripetal is the best response to treatment. Centripetal phenomenon can reduce pain and restore patients' ability to work. In recent years, it has also been recognized by Chinese patients and doctors. In clinical practice, we should use appropriate body position extension, continuous extension, extension position rotation relaxation, bending position rotation relaxation, bending position rotation, extension position rotation, and flexible sensitive position.

*(5) Joint Mobilization.* The general activity is based on the biomechanical principle of joint movement. Small movement is carried out on the joint surface to cause large joint movement. In the face of stiff joints, limited movement, pain, or numbness, it is beneficial to relieve muscle spasm and pain by making average rhythm and repetitive passive activities. The range of motion is to restore the normal motion of the joint, and the mode of motion is passive normal motion and passive auxiliary motion. Vibration technology and continuous intra-articular motion technology are most widely used in clinical practice [15].

*(6) Core Strength Training.* Core stability is the central link of sports training, which also has an important protective effect on human bones. Joints and muscles can maintain the balance of the waist. The main movement of resistance is to control spinal instability and relieve back pain and abdominal muscles by strengthening the muscle strength of lower back muscles and muscles. Only by keeping the right balance of abdominal and back muscles can we keep a good posture and keep the stability of spinal cord. In clinical practice, sports, fitness ball, and air cushion are used in bridge practice, bridge practice, smoking practice, body bending, knee balance training, etc. Low muscle function exercise is also considered to be an effective way to treat low back pain, which can significantly improve lower back pain and lower back muscle strength [16, 17]. In clinical work, doctors often support the functional exercise of lower back muscles in patients with low back pain to enhance muscle strength and repair or strengthen the stability of spine. After daily exercise is stable, healthy people can also increase the strength of back and back muscles to improve their ability to control spinal movement and prevent injury.

*(7) Rehabilitation Engineering.* For patients with severe back pain and poor lumbar stability, they should wear braces, strengthen and protect the spine, limit movement, stabilize disease, reduce pain, reduce the weight of vertebrae, and improve their daily ability. In clinical practice, we often think that patients with acute spinal cord injury should wear a brace, but not for a long time, so as not to weaken the strength of lumbar muscles, make the lumbar system worsen, and make patients have mental dependence.

*(8) Psychotherapy.* Most patients with low back pain have psychological and emotional effects; depression and anxiety are common adverse emotional reactions of LBP patients, and the impact on the occurrence and development of LBP has attracted more and more attention. Early psychological intervention and self-exercise can better treat and prevent low back pain [18]. We should actively help patients to eliminate or reduce the burden of thinking, psychological pain and enhance the confidence of treatment.

### 2.4. Preparation of Bismuth Tungstate Nanomaterials

#### 2.4.1. Solid-Phase Sintering

Solid-phase sintering is a relatively early method to prepare Bi_2_WO_6_ powder. In the past, this method was mostly used to prepare Bi_2_WO_6_ powder. This method is realized by directly burning the oxides containing Bi and W elements or their salts at high temperature. This method is simple to operate, but usually needs to react at a higher temperature, which is not conducive to energy conservation. Moreover, due to the larger particle size and smaller specific surface area of the catalyst prepared by this method, the pollutants attach less on the catalyst surface, Therefore, the photocatalytic activity is not high [19]. Therefore, in recent years, with the development and progress of science and technology, solid methods have been basically eliminated.

#### 2.4.2. Precipitation Method

In the method, the metal salt solution reacts with the settling agent to wash, filter, etc., sediment that produces the final product. The equipment needed by the method is relatively simple and easy to use, which can be used in large-scale industrial production. However, the products produced by this method only use milling process to produce crystal materials. On the one hand, in the process of processing, a lot of energy consumption is needed in the burning process, which is easy to cause product accumulation and make the particle size larger, which is not conducive to improving the photocatalytic performance of the products.

#### 2.4.3. Sol-Gel Method

As a method of synthesizing inorganic materials under mild conditions, sol-gel method plays an important role in soft chemical composition [20, 21]. In this method, a series of chemical reactions of inorganic salt in organic solvent form a substance similar to colloid, which can be dried and ground to obtain the required powder material. This method has some advantages and disadvantages: the physical and chemical properties of the obtained sol are relatively uniform and stable; the reaction can generally be carried out at room temperature; however, the cost of the raw materials used is more, and if people contact for a long time, it will cause health hazards; secondly, the preparation steps are more, and the reaction time is too long; finally, the large shrinkage will occur in the later treatment process. Therefore, considering the principle of simple operation, this method is not recommended.

#### 2.4.4. Sonochemistry

Due to the principle of acoustic cavitation, under the influence of ultrasound, the formation and development, the collapse of micro bubble core in liquid and a series of physical and chemical reactions are caused. It can quickly collect and release the energy released by the sound field, which provides solutions for some chemical reactions that are impossible or difficult to occur under normal conditions. Ultrasonic synthesis can be used for the successful preparation of Bi_2_WO_6_ nanospheres, and its development mechanism is mainly affected by this method [22, 23]. The biggest advantage of ultrasonic chemical composition method is that it does not need solvent, and the time can be shortened to dozens of minutes, but the biggest disadvantage is that the reaction is not easy to control, horizontal reaction occurs, and the microwave reactor is expensive, so it can only be used on a small scale in the laboratory, and it is difficult to produce ionic liquid on a large scale. Therefore, it has not been widely used in powder manufacturing.

#### 2.4.5. Hydrothermal Method

Hydrothermal method is one of the methods of liquid-phase chemical synthesis. It uses high temperature and high pressure conditions to make the substances that cannot be synthesized under normal temperature react and reduces the activation energy of the reaction through external action so as to grow crystals in a closed environment. It is widely used in the preparation of ultrafine particles, inorganic films, and microporous materials [24]. Hydrothermal method can directly prepare the powder with good crystallinity, avoiding the agglomeration caused by high-temperature sintering; the preparation process is relatively simple; by changing the hydrothermal conditions, the grain size and morphology of the product can be controlled, so the performance of the product can be changed, so it has become a mature method for preparing nano/micro powder. The hydrothermal method has the advantages of low cost, simple process, and low reaction temperature. However, the equipment has high requirements, difficult technology, and poor safety performance. Even so, hydrothermal method has become a common method for preparing Bi_2_WO_6_.

#### 2.4.6. Solvothermal Method

Solvothermal method is an extension of traditional hydrothermal method. It is different from hydrothermal method. The solvent it uses is an organic solvent rather than water. One of the advantages of using organic solvent as reaction medium is that it can make the dispersibility of the product and the boiling point of organic solvent better, usually lower, so the reactivity is increased, so the temperature required for the reaction becomes lower, which helps to save energy. However, the organic solvent used in solvothermal method will cause the instability of the system, which is prone to explosion and other dangerous accidents. In addition, some organic solvents are toxic and not good for the body, so from the perspective of environmental protection and health, this method is not recommended.

#### 2.4.7. Microemulsion Method

Two immiscible solvents are mixed to form a milk-like solution, in which microbubbles are generated, the reagents are combined to form crystalline nuclei, and then heat treatment is carried out. The method of preparing nanoparticles in this way is called microemulsion method. Microemulsion systems are usually solvents, water, surfactants, and cosurfactants. The ambiguous molecules in surfactants can divide the incompatible continuum into micro regions (nanoscale). The method is used to prepare nanoparticles, and the required experimental device is simple, consumes low energy, and is convenient to operate. The disadvantage is that the molecular gap of the material is large. As a microreactor, the reagents in the microreactor can react to form solid particles. It is generally believed that the reaction mechanism of the micro coating method is the formation of microbubbles using instantaneous negative phase voltage [25]. Because the micro coating method can accurately control the size and thermodynamic stability of nanoparticles, and by controlling the formation and development of nanoparticles in the micronucleus, a certain concentration structure may be formed, and a layer of nanoparticles with surface activity is wrapped on the surface. The particle interface obtained by this method is better. If teen-80 is used as a surfactant, *n*-butanol as a cosurfactant and *n*-heptane as the oil phase; then double solution (NO_3_) is added to the dilute nitric acid through stirring to obtain microemulsion and Bi_2_WO_6_ photocatalyst.

## 3. Experiments

### 3.1. Preparation and Characterization of Experimental Samples

In this experiment, bismuth tungstate nanomaterials were prepared by hydrothermal method. The hydrothermal method can directly prepare powders with good crystallinity, avoiding agglomeration caused by high-temperature sintering. The preparation process is relatively simple. Hydrothermal crystal growth mainly uses the temperature difference between the upper and lower solutions of the high-temperature reactor to make the solution in the reactor produce strong convection and never bring the saturated solution in the high-temperature zone to the low-temperature zone with seed crystals to form supersaturated solution. Therefore, according to the classical crystal growth theory, crystal growth under hydrothermal conditions includes the following steps:

1. The precursor dissolves in the hydrothermal medium and enters the solution in the form of ions and molecular groups (dissolution stage).
2. Due to the very effective thermal convection and the concentration difference between the dissolution zone and the growth zone, these ions, molecules, or ion clusters are transported to the growth zone (transport stage).
3. Adsorption, decomposition, and desorption of ions, molecules, or ion groups at the growth interface.
4. The movement of adsorbed material on the interface.
5. Crystallize.

By changing the hydrothermal conditions, the crystal size and morphology of the products can be controlled; thus, the properties of the products can be changed, so it has become a mature method for preparing nano/micro powders. The hydrothermal method has the advantages of low cost, simple process, and low reaction temperature. The hydrothermal method has become a common method for preparing Bi_2_WO_6_. The raw materials are Bi (NO_3_)_3._5H_2_O, analytical pure Na_2_WO. 2H_2_O, and trimethyl bromide (CTAB).

### 3.2. Test Steps

The experimental steps are as follows: weigh 2.419 g Na_2_WO.2H_2_O and 4.851 g Bi (NO_3_)_3_.5H_2_O in 100 ml of desalted water, adjust the pH value of the solution with nitric acid and sodium hydroxide, stir for 30 min, and add a certain amount of CTAB concentration of 0, 0.02, 0.04, 0.06, and 0.08, respectively, in mol/L; the solution has been transferred to the polytetrafluoroethylene reaction tank (the filling rate is about 75%), and the reaction is carried out in OC (organic carbon) for 24 hours and then cooled naturally at room temperature to obtain light yellow sediment. Wash with water and ethanol several times, dry and sample at 80-8451 constant temperature. Using Shimadzu X-ray reflector Shimadzu XRD-7000, using CuKa radiation, *l* = 15406 nm, 40 kV tube voltage, and 30 mA tube current, the phase structure was analyzed, the grade detection was carried out, the step length was 0.02, and the step scanning time was 2S. The morphology of Bulgarian tungsten material Jeol-2010f (TEM) transport was observed by using HITACHI s-4800 electron microscope and electron microscope.

### 3.3. Photocatalytic Performance

Prepare the hydrochloric acid aqueous solution with the concentration of 100 mg/L, weigh 0.20 g bismuth tungstate sample, disperse it in 100 ml hydrochloric acid aqueous solution, and adjust the pH value of the system to 2; after ultrasonic dispersion for 10 minutes, irradiate it with low beam sunlight bulb; take out 5 ml of the filtered solution regularly and quantitatively. At the same time, a concentration absorption curve is formed to calculate the residual concentration ratio or elimination rate: CT/C0, where CT and C0 are reaction time *t* and initial hydrochloric acid solution concentration, respectively. During the experiment, the changes of color, temperature, and precipitate of the solution were recorded. Carry out many experiments to eliminate the chance of the experiment.

## 4. Discussion

### 4.1. Effect of Ph Value on the Structure and Morphology of Samples

Figure 2 shows the XRD patterns of bismuth tungstate samples obtained by hydrothermal method at different pH values (3, 5, 7, 9, and 11, resp.) without adding surfactants.

It can be seen from Figure 2 that the XRD standards of bismuth tungstate samples collected in pH 3 and 5 are the same, with peak value, indicating that the samples are clean Bi_2_WO_6_; in pH = 7, in addition to the peak resolution of Bi_2_WO_6_ phase, there are also small equipartial peaks in the samples; when the pH value increases to 9, the resolution peak of Bi_2_WO_6_ phase is very sharp, and the resolution peak of heterophase is also very obvious. Once the phase is evaluated as cubic Bi_3.84_W_Q.16_O_6.24_, the sample produced under these conditions is a biphasic mixture of Bi_2_WO_6_ and Bi_3.84_W_Q.16_O_6.24_; when the pH value increases to 11, the resolution peak of Bi_2_WO_6_ disappears completely, and only the deflection peak of Bi_3.84_W_Q.16_O_6.24_ exists, indicating that the sample is pure Bi_3.84_W_Q.16_O_6.24_. It can be seen from the above analysis that the value of *R* in the reaction system has a great influence on the structure of the sample. At low pH (3∼5), the sample is pure Bi_2_WO_6_. The increase of pH value of the reaction system is conducive to the formation of Bi_3.84_W_Q.16_O_6.24_. At high pH ( > 11), 24 phases appeared in the reaction products, Bi_2_WO_6_ phase disappeared, and only pure Bi_3.84_W_Q.16_O_6.24_ appeared. The products and morphology under different pH values are shown in Table 1.

From the observation of Figures 3(a) and 3(b), it can be seen that when the pH value is low (3–5), the samples are all dispersed nano blade structure with irregular edge. When the pH value increases to 7, the nano leaves tend to change from irregular shape to square, and the edges become slightly clean. When the pH value is 9, a large sample of a structure similar to a square plate appears. In addition, some octahedral nanoparticles have also appeared. The enlarged scanning of the square leaf structure is shown. Obviously, the structure of the square leaf in the sample is relatively normal, and the side length is about 200–300 nm. When the pH value increased to 11, the nano desulfurization structure disappeared completely at low pH, and only octahedral nanoparticles with very smooth surface were found in the samples. According to the observation in Figures 3(a) and 3(b), different pH values in the reaction system lead to the appearance of bismuth tungstate samples with different structures, which in turn leads to different morphologies of the samples. At low pH, the sample is Bi_2_WO_6_. With the increase of pH value, the samples were transformed into Bi_3.84_W_Q.16_O_6.24_.

The composition of Bi_2_WO_6_ crystal elements is shown in Figure 4.

The appearance of W-Bi nanomaterials with different morphology is due to the different solubility of WO_6_ and Bi_2_O_2_ in different pH solutions. At the pH value of 3–5, the OH^−^ concentration in the solution is far lower than that of H^+^, which inhibits the hydrolysis of Bi_2_O_2_, reduces the growth rate of Bi_2_WO_6_ crystal, improves the nucleation and aggregation rate of Bi_2_WO_6_, and creates a leaf-like structure. When the pH value increases to 7, the concentration of OH^−^ and H^+^ in the solution is the same, and the hydrolysis degree of Bi_2_O_2_ is moderate, but there are more WO_6_ dissolved in the solution, and the amount of WO_6_ used for Bi_2_WO_6_ dissolution is reduced, so the dissolution rate of Bi_2_WO_6_ is also limited. At present, the preparation speed of Bi_2_WO_6_ nanospheres has not been significantly improved. When the pH value increased to 9, the hydrolysis reaction of Bi_2_O_2_ was enhanced, and the solubility of WO_6_ in alkali solution was higher. Therefore, Bi_2_WO_6_ crystal was prepared with less WO_6_, and the second phases Bi_2_WO_6_ and Bi_3.84_W_Q.16_O_6.24_ of Bi_3.84_W_Q.16_O_6.24_ were obtained. When the pH value increases to 11, the solubility of WO_6_ is higher. Only a small amount of WO_6_ is used to form crystals, which is inhibited by the isotropic development of crystals, so Bi_3.84_W_Q.16_O_6.24_ in octahedron form becomes the main phase.

### 4.2. CTAB Concentration Effect on Product Morphology

When the double surfactant material is added, different surfactants can be used for sampling, which have different forms. Bi_2_WO_6_ material was prepared with PVP as surfactant, and chrysanthemum Bi_2_WO_6_ material was obtained. Cetyltrimethylammonium bromide (CTAB), as a common surfactant, is widely used in the morphology control of nanomaterials, but the effect of CTAB on the morphology of Bi_2_WO_6_ has not been reported. CTAB is a kind of surfactant. Five groups of CTAB with different concentrations of 0, 0.02 mol/L, 0.04 mol/L, 0.06 mol/L, and 0.08 mol/L were added to the reaction system to investigate the effect of CTAB concentration on the morphology of the product.

In the absence of CTAB, the sample has a nanostructure similar to the result in Figure 2(b). When 0.02 mol/l CTAB was added into the reaction system, the morphology of the sample changed. Although it is also a nano leaf structure, it is interconnected. When the CTAB concentration is 0.04 mol/L, the nanotubes are stacked together under the action of surfactant. When the concentration of CTAB increased to 0.06 mol/L, the self-assembled nanocomposites tended to be petal like. When the concentration of CTAB is 0.08 mol/l, there is a petal-like structure composed of several nanoflakes. The above results show that the addition of CTAB can affect the morphology of Bi_2_WO_6_, which tends to self-assembly under the influence of thin-layer mycelium molecules and finally forms petal like structure. The product morphology at different CTAB concentrations is shown in Table 2.

### 4.3. Photocatalytic Performance

The pain caused by lactic acid is always a difficult problem in the treatment of lumbar disc herniation. Therefore, hydrochloric acid was used as the experimental object to study the photocatalytic degradation of bismuth tungstate samples with different structures and morphologies under different pH values. The results are shown in Figure 5.

It can be seen from Figure 5 that the maximum absorption peak of hydrochloric acid solution is Lmax = 538 nm, which is caused by the structural transformation of hydrochloric acid. After about 15 minutes, the hydrochloric acid solution was absorbed close to 0, which indicated that hydrochloric acid was basically completely degraded, indicating that Bi_2_WO_6_ nanospheres prepared under pH 3 had obvious catalytic degradation effect on hydrochloric acid under visible light. According to the light absorption curve of the coexisting samples Bi_2_WO_6_ and Bi_3.84_W_Q.16_O_6.24_ on the degradation of hydrochloric acid solution, the time of complete degradation of hydrochloric acid is extended to about 45 minutes, and the degradation rate is reduced compared with the clean samples of Bi_2_WO_6_, indicating that there is Bi_3.84_W_Q.16_O_6.24_ phase in the sample, and the photodegradation effect is not as good as that of pure Bi_2_WO_6_ phase.

## 5. Conclusions

In this paper, bismuth tungstate nanomaterials with different morphologies were obtained by adjusting the pH value or CTAB concentration of the solution by hydrothermal method. The experimental results show that when the pH value is low, the sample is Bi_2_WO_6_ nanoflake, and the content of bi3.84wq.16o6 increases with the increase of pH value. At high pH, the pure-phase octahedral nanoparticle appears. The sample is pure octahedral nanoparticle Bi_3.84_W_Q.16_O_6.24_, and the surfactant CTAB is in the reaction solution The different concentrations in the sample also affect the morphology of Bi_2_WO_6_. With the increase of CTAB concentration, Bi_2_WO_6_ samples were self-assembled into petal-like structure. Bi_2_WO_6_ phase sample has a good catalytic degradation effect on hydrochloric acid solution and a good medical effect on the rehabilitation treatment of lumbar disc herniation.

In addition, combined with the basic methods to treat lumbar disc herniation, XRD and FESEM analyses of bismuth tungstate nanomaterials with different structures and morphologies were carried out, and the structure and morphologic characteristics of the samples were analyzed, and the effect of rehabilitation training for the patients with lumbar disc herniation was studied. The experimental results are in line with the expectations and can be applied to clinical experimental studies.

In this paper, the photocatalysis of bismuth tungstate nanomaterials with different structures and shapes under different pH values and CTAB concentrations is studied. The results show that the sheet bismuth tungstate nanomaterials have the best catalytic effect on hydrochloric acid, while hydrochloric acid and lactic acid have similar properties, indicating that the sheet bismuth tungstate nanomaterials also have the same effect on the lactic acid produced by human body, reflecting the fact that the sheet bismuth tungstate nanomaterials have the same effect on lumbar disc protrusion. The rehabilitation treatment has medical value.

## Figures and Tables

**Figure 1:** Effect of excessive displacement of some parts of the spine.

**Figure 2:** XRD patterns of bismuth tungstate samples prepared at different pH values.

**Figure 3:** FESEM photos of bismuth tungstate samples prepared at different pH values.

**Figure 4:** Schematic diagram of Bi_2_WO_6_ crystal element composition.

**Figure 5:** UV-Vis absorption curve of bismuth tungstate photocatalytic degradation of hydrochloric acid solution and the relationship between hydrochloric acid removal rate and time.

**Table 1:** Products and morphology at different pH values.

PH value	3	5	7	9	11
Product	Bi_2_WO_6_	Bi_2_WO_6_	Bi_2_WO_6_ Bi_3.84_W_Q.16_O_6.24_ (trace)	Bi_2_WO_6_ Bi_3.84_W_Q.16_O_6.24_	Bi_3.84_W_Q.16_O_6.24_

Morphology	Scattered nanoflakes	Scattered nanoflakes	The trend of changing from irregular shape to square; the edge becomes a little neat	Square sheet	Octahedral shape

**Table 2:** Product morphology at different CTAB concentrations.

CTAB concentration	0 mol/L	0.02 mol/L	0.04 mol/L	0.06 mol/L	0.08 mol/L
Morphology	Nanosheet	Crosslinked nanoflake	Laminated nanosheet	Assembling nanoflakes	Petal shaped

## Data Availability

No data were used to support this study.
